The article "Long non-coding RNA SNHG16 regulates cell behaviors through miR-542-3p/HNF4α axis via RAS/RAF/MEK/ERK signaling pathway in pediatric neuroblastoma cells" was retracted in 2024. Reasons: plagiarized images; duplicated images; overlap with other authors' work; overlap with earlier publications.

# Long non-coding RNA SNHG16 regulates cell behaviors through miR-542-3p/HNF4α axis via RAS/RAF/MEK/ERK signaling pathway in pediatric neuroblastoma cells

**DOI:** 10.1042/BSR20200723

**Published:** 2020-05-26

**Authors:** Defeng Deng, Shuangjie Yang, Xiang Wang

**Affiliations:** Department of Hematology, Kaifeng Children’s Hospital, Kaifeng, Henan, China

**Keywords:** HNF4α, miR-542-3p, neuroblastoma, RAS/RAF/MEK/ERK signaling pathway, SNHG16

## Abstract

Neuroblastoma (NB) is an extracranial solid tumor in children with complex mechanism. Increasing reports indicated that long non-coding RNA (lncRNA) small nucleolar RNA host gene 16 (SNHG16) account for the pathogenesis of NB. Nevertheless, the precise functions of SNHG16 needed to be further exposed in NB progression. Our data revealed that SNHG16 and hepatocyte nuclear factor 4 α (HNF4α) were up-regulated, but miR-542-3p was down-regulated in NB. Knockdown of SNHG16 or HNF4α could impede cell proliferation, migration, invasion, and epithelial–mesenchymal transition (EMT) *in vitro*. Interestingly, the role of SNHG16 detetion in cell behaviors was rescued by HNF4α overexpression in NB cells. Mechanically, SNHG16 modulated the progression of tumor growth via miR-542-3p/HNF4α axis in NB. Also, SNHG16 knockdown inactivated rat sarcoma/effector of RAS/mitogen-activated extracellular signal-regulated kinase/extracellular regulated protein kinases (RAS/RAF/MEK/ERK) signaling pathway through HNF4α. Therefore, SNHG16/miR-542-3p/HNF4α axis modified NB progression via RAS/RAF/MEK/ERK signaling pathway, might highlight a novel therapeutic approach for NB.

## Introduction

Neuroblastoma (NB) is a typical solid tumor characterized by extracranial injury. After statistics, researchers showed that the death from NB occupies ∼15% of all deaths from cancer in children [1]. Besides, more than 90% of NB patients are diagnosed when the age less than 10 years [2]. The tumor of NB shows widely enigmatic behaviors, such as the spontaneously regresses in infants, and the continuous proliferation in children when the age over than 1 year [3,4]. Although the persistent development of the therapeutic approaches, the 5-year survival rate of NB patients remains disappointingly low after disease relapse [5]. Hence, it is necessary to search for efficient therapeutic strategies for NB treatment.

Currently, numerous long non-coding RNAs (lncRNAs; over than 200 nucleotides in length) have been found to exist in various tumors [6], such as breast cancer [7], colorectal cancer [8], and NB [9]. In addition, the expression of lncRNAs in tumor tissues is obviously different from the non-tumor masses. These aberrantly expressed lncRNAs may go in for the transcription and post-transcriptional translation [10]. Previous works revealed that lncRNAs acted as critical roles in the regulatory mechanism of multiple cancers. Moreover, lncRNAs frequently functioned as competing endogenous RNA (ceRNA) to regulate gene expression, thereby dysregulating cell functions [11]. Besides, lncRNA small nucleolar RNA host gene 16 (SNHG16) has been reported to participate in the process of diverse diseases, including hepatocellular carcinoma [12,13] and NB [9]. Based on the earlier researches, we further investigated the role of SNHG16 in NB development.

The article "Long non-coding RNA SNHG16 regulates cell behaviors through miR-542-3p/HNF4α axis via RAS/RAF/MEK/ERK signaling pathway in pediatric neuroblastoma cells" was retracted in 2024. Reasons: plagiarized images; duplicated images; overlap with other authors' work; overlap with earlier publications.

Over the past decades, increasing researchers discovered some types of non-coding RNAs (ncRNAs). Of which microRNAs (miRNAs, 20–25 nucleotides in length) belong to ncRNAs, and they have been recognized as novel biomarkers and therapeutic targets for cancers [14]. Most often, miRNAs are target genes of lncRNAs, such as SMHG16 acts as an oncogenic factor to regulate pancreatic cancer growth by sponging miR-218-5p [15]. Furthermore, the tumor-suppressive or oncogenic role of miRNAs depends on a series of targeted mRNA, the incomplete complementation between miRNAs and mRNAs can dysregulate the expression of the targeted genes [16]. MiR-542, as a general member of miRNAs, has been manifested to be down-regulated in several tumors [17,18]. And the two isoforms of miR-542-3p and miR-542-5p are related to the prognosis, and both of them function as tumor suppressors in NB pathogenesis and progression [19,20]. Herein, we focused on the underlying role of miR-542-3p in NB development.

Until now, hepatocyte nuclear factor 4 α (HNF4α) is a highly conserved transcription gene, it has been proved to be involved in the development of cancerous diseases [21]. We hypothesized that HNF4α was a target gene of miR-542-3p, the potential role of HNF4α was needed to be explored. Additionally, rat sarcoma/effector of RAS/mitogen-activated extracellular signal-regulated kinase/extracellular regulated protein kinases (RAS/RAF/MEK/ERK) signaling pathway is associated with tumorigenesis. For example, miR-30a functioned the antitumor role via repressing RAS/RAF/MEK/ERK pathway [22].

In the paper, we researched the expression patterns of SNHG16, miR-542-3p, and HNF4α in pediatric NB tissues and cell lines, and the functions of them in cellular behaviors were exposed by the subsequent assays.

## Materials and methods

### Clinical samples and cell culture

Specimens (30 of NB tissues and 30 of adjacent non-tumor tissues) were received from NB patients who ranged in age from 8 months to 8 years. The patients were diagnosed and treated in Kaifeng Children’s Hospital. The study was approved by the Ethics Committees of Kaifeng Children’s Hospital, and the written informed consents were obtained from all the participant

NB cells (SKNBE-2, SK-N-SH) and human embryonic kidney 293 cells (HEK293) were obtained from American Type Culture Collection (ATCC), and the other NB cells (LAN-5) were purchased from FENGHUI SHENGWU Co., Ltd (Hunan, China). Of which SKNBE-2 were grown in the mixture of equal Eagle’s Minimum Essential Medium (EMEM) and F12 medium (Thermo Fisher Scientific, Rockford, IL, U.S.A.), LAN-5 cells and HEK293 cells were maintained in EMEM. The above cell culture mediums were supplemented with fetal bovine serum (FBS; 10%, Gibco, Carlsbad, CA, U.S.A.), penicillin (100 U/ml; Gibco), and streptomycin (100 mg/ml; Gibco). Then, cells were cultured in a 5% CO_2_-humidified incubator.

The article "Long non-coding RNA SNHG16 regulates cell behaviors through miR-542-3p/HNF4α axis via RAS/RAF/MEK/ERK signaling pathway in pediatric neuroblastoma cells" was retracted in 2024. Reasons: plagiarized images; duplicated images; overlap with other authors' work; overlap with earlier publications.

### Quantitative real-time polymerase chain reaction assay

For assay of the level of miR-542-3p, miRNA was extracted from tissues (NB and non-carcinoma tissues) and cells (SKNBE-2, SK-N-SH, LAN-5, and HEK293) using miRVana kit (Ambion, Austin, TX, U.S.A.). Then, One-Step Primescript miRNA cDNA synthesis kit (Takara, Dalian, China) was adopted to conduct a transcription reaction. The relative expression level of miR-542-3p was quantified and normalized to U6. For analysis of the expression of lncRNA and mRNA, total RNA was separated and extracted utilizing TRIzol (Invitrogen, Carlsbad, CA, U.S.A.), and M-MLV reverse transcriptase (Promega, Madison, WI, U.S.A.) was administrated to form cDNA according to standard manuals. Subsequently, cDNA template, relative primers, and AceQ qPCR SYBR Green Master Mix (Vazyme, Nanjing, China) were subjected to a real-time polymerase chain reaction. The relative expression of SNHG16 and HNF4α were standardized to glyceraldehyde-3-phosphate dehydrogenase (GAPDH). All the primers were listed: SNHG16 (forward: 5′-GTTCCTCTAAGTAATCGCCATGCGTTCT-3′, reverse 5′-CATTTCAGTTTACAATCCTTGCAGTCCC-3′); miR-542-3p (forward: 5′-TGTGACAGATTGATAACT-3′, reverse 5′-GTGCAGGGTCCGAGGT-3′); HNF4α (forward: 5′-CATGGACATGGCCGACTACAG-3′, reverse 5′-CGTTGAGGTTGGTGCCTTCTGA-3′); GAPDH (forward: 5′-CAGCTAGCCGCATCTTCTTTT-3′, reverse 5′-GTGACCAGGCGCCCAATAC-3′); U6 (forward: 5′-CTCGCTTCGGCAGCACA-3′, reverse 5′-AACGCTTCACGAATTTGCGT-3′).

### Western blot

The operation of the Western blot was referenced the previous instructions [23]. Briefly, the protein was combined with primary antibodies, and the corresponding secondary antibody was applied to bind to the unique antibody. In the end point, the special protein was visualized via a Visualizer Western Blot Detection Kit (Millipore, Bedford, MA, U.S.A.). The primary antibodies were introduced as follows: HNF4α (ab201460, 1:1000), E-cadherin (ab76055, 1:1000), Vimentin (ab8979, 1:1000), N-cadherin (ab18203, 1:500), phospho-RAF (p-RAF; ab173539, 1:3000), GAPDH (ab8245, 1:5000), RAS (3965, 1:1000), phospho-ERK (p-ERK; 9101, 1:1000), and phospho-MEK (p-MEK; 9154; 1:1000). Of which HNF4α, E-cadherin, Vimentin, N-cadherin, p-RAF, and GAPDH were purchased from Abcam (Cambridge, MA, U.S.A.), RAS, p-ERK, and p-MEK were obtained from Cell Signaling Technology (Boston, MA, U.S.A.).

The article "Long non-coding RNA SNHG16 regulates cell behaviors through miR-542-3p/HNF4α axis via RAS/RAF/MEK/ERK signaling pathway in pediatric neuroblastoma cells" was retracted in 2024. Reasons: plagiarized images; duplicated images; overlap with other authors' work; overlap with earlier publications.

### Transient transfection

Small interfering RNA (siRNA) against SNHG16 (si-SNHG16) and HNF4α (si-HNF4α), siRNA negative control (si-NC), short hairpin RNA (shRNA) against SNHG16 (sh-SNHG16), shRNA negative control (sh-NC), overexpression vectors of SNHG16 (pcDNA-SNHG16) and HNF4α (pcDNA-HNF4α), as well as their control constructed by pcDNA3.1 vector (pcDNA) were designed and synthesized in Ribobio (Shanghai, China). Furthermore, miR-542-3p mimic (miR-542-3p) and its blank control (miR-NC) were constructed from Ribobio. All the sequences were introduced into SKNBE-2 and SK-N-SH cells using Lipofectamine 2000 reagent (Invitrogen) based on the specifications. Meanwhile, lentivirus-mediated sh-SNHG16 or sh-NC was introduced into SKNBE-2 cells to form stably transfected cells.

### Cell proliferation detection

3-(4,5-dimethylthiazol-2-yl)-2,5-diphenyl-tetrazolium bromide (MTT) was conducted to examine the ability of cell proliferation in NB cells. First, the transfected cells were seeded into a 96-well plate, after transfection for 0, 24, 48, or 72 h, the old medium was abandoned, and 20 µl MTT reagent was supplemented into each well, and cells were continuously incubated at 37°C for 4 h. Then, the formative precipitate was dissolved via adding 200 µl of dimethyl sulfoxide (DMSO; Sigma, St. Louis, MO, U.S.A.). At last, the absorbance of lysates was estimated via a microplate reader at 490 nm.

### Transwell assay

In the cell migration assay, equal numbers of NB cells (non-transfected and stably transfected) were loaded into the upper chamber with serum-free media. At the same time, the complete medium was added into the lower chamber. Then, the cells were incubated in 37°C with 5% CO_2_ for 24 h. The cells remained in the upper chamber were erased using cotton swabs, and the migrated cells were stained with Crystal Violet (0.1%; Sigma). The cells were photographed at least in five random fields. For cell invasion assay, the upper chamber was pre-coated Matrigel (BD Bioscience, San Jose, CA, U.S.A.) before cells were seeded on to the surface, the following protocol was in line with cell migration assay.

### Dual-luciferase reporter assay

The common fragments containing the binding sites between miR-542-3p and SNHG16 or HNF4α were amplified and inserted into the luciferase promoter vector of pGL3 (Promega), then luciferase reporters were formed, including SNHG16 WT and HNF4α 3′UTR-WT. As the controls, the mutant nucleotides of the above binding sites were designed to construct mutant reporters (SNHG16 MUT and HNF4α 3′UTR-MUT). After that, SKNBE-2 and SK-N-SH cells were co-transfected with wild-type or mutant reporters and miR-542-4p or miR-NC, respectively. Cells were harvested at 48 h post-transfection, and the firefly and *Renilla* activities were determined using a dual-luciferase reporter assay kit (Promega) in the light of standard protocols.

The article "Long non-coding RNA SNHG16 regulates cell behaviors through miR-542-3p/HNF4α axis via RAS/RAF/MEK/ERK signaling pathway in pediatric neuroblastoma cells" was retracted in 2024. Reasons: plagiarized images; duplicated images; overlap with other authors' work; overlap with earlier publications.

### *In vivo* xenograft model

BALB/c nude mice were obtained from Shanghai Laboratory Animal Center Co., Ltd. (Shanghai, China), all the mice were raised and operated in accordance with the Institutional Animal Care and Use Committee of Kaifeng Children’s Hospital. And all animal experiments were carried out at Kaifeng Children’s Hospital. For tumor growth assay, mice were divided into two groups (*n*=5/group) randomly, the stably transfected SKNBE-2 cells were diluted in 200 µl of phosphate buffered saline (PBS; Gibco) and then injected into the left flank of nude mice subcutaneously. The tumor volume was measured every 4 days for six times at 7 days post-injection. We calculated the tumor volume according to the formula: volume (V) = length (L) × width^2^ (W^2^) × 0.5. After injection for 27 days, mice were killed by cervical dislocation after anesthesia with isoflurane (2%), and the tumor tissues were fetched and weighed.

### Statistical analysis

The data were exhibited as mean ± standard error of the mean (SEM). Comparisons between controls and treated groups were performed utilizing either Student’s *t* test (for two-group) or one-way ANOVA (for multiple groups). The statistical difference was defined as *P*-value less than 0.05.

## Results

### SNHG16 and HNF4α were up-regulated in NB tissues and cell lines

First, the level of SNHG16 in NB tissues and cell lines were detected. As shown in Figure 1A,B, the level of SNHG16 was notably higher in NB tissues and cell lines compared with the corresponding non-tumor tissues and cells. Then we examined the mRNA and protein levels of HNF4α, the findings indicated that both mRNA and protein levels of HNF4α were remarkably reinforced in NB tissues and cell lines (Figure 1C–F). Moreover, the correlation between HNF4α and SNHG16 was investigated, quantitative real-time polymerase chain reaction (qRT-PCR) analysis demonstrated that SNHG16 level was positively related to HNF4α level (Figure 1G). All the data exposed that the aberrant expression of SNHG16 and HNF4α might be involved in the progression of NB.

The article "Long non-coding RNA SNHG16 regulates cell behaviors through miR-542-3p/HNF4α axis via RAS/RAF/MEK/ERK signaling pathway in pediatric neuroblastoma cells" was retracted in 2024. Reasons: plagiarized images; duplicated images; overlap with other authors' work; overlap with earlier publications.

**Figure 1:** SNHG16 and HNF4α were up-regulated in NB tissues and cell lines (**A,B**) The level of SNHG16 in (A) NB tissues and (B) cell lines was evaluated using qRT-PCR. (**C**–**F**) The (C,E) mRNA and (D,F) protein levels of HNF4α in NB tissues and cell lines were examined via qRT-PCR and Western blot assays, respectively. (**G**) qRT-PCR was carried out to analyze the correlation between SNHG16 level and HNF4α level. *P<0.05.

### SNHG16 deficiency hindered cell proliferation, migration, invasion, and epithelial–mesenchymal transition in NB cells

Given the unusual expression of SNHG16 in NB tissues, we aimed to explore the biological role of SNHG16 in the pathogenesis of NB. First, si-SNHG16 or si-NC was transfected into SKNBE-2 and SK-N-SH cells, qRT-PCR analysis displayed that the knockdown efficiency could live up to the expectation (Figure 2A). Next, the effect of si-SNHG16 on cell proliferation was estimated using MTT assay, the results manifested that cell proliferation was particularly hindered via SNHG16 detetion *in vitro* (Figure 2B,C). Simultaneously, transwell analysis discovered that the capacities of mobility and invasiveness were both reduced in SKNBE-2 and SK-N-SH cells (Figure 2D,E). Meanwhile, the expression levels of E-cadherin, N-cadherin, and Vimentin were assessed using Western blot, the high expression of E-cadherin, and the low expression of N-cadherin and Vimentin showed the suppressive impact of SNHG16 silencing on epithelial–mesenchymal transition (EMT) (Figure 2F–I). These findings meant that knockdown of SNHG16 significantly constrained cell proliferation, migration, invasion, and EMT in NB cells.

**Figure 2:** SNHG16 deficiency hindered cell proliferation, migration, invasion, and EMT in NB cells (**A**) The knockdown efficiency of si-SNHG16 in SKNBE-2 and SK-N-SH cells was determined. (**B,C**) The effect of si-SNHG16 on cell proliferation was identified by MTT assay *in vitro*. (**D,E**) Transwell assay was performed to detect the capacity of mobility and invasiveness in SKNBE-2 and SK-N-SH cells. (**F**–**I**) Western blot assay was employed to estimate the expression levels of E-cadherin, N-cadherin, and Vimentin in transfected SKNBE-2 and SK-N-SH cells. *P<0.05.

### HNF4α knockdown restrained cell proliferation, migration, invasion, and EMT *in vitro*

To gain insight into the function of HNF4α in NB pathogenesis, we established the knockdown vector of HNF4α, and then si-HNF4α or si-NC was introduced into SKNBE-2 and SK-N-SH cells. qRT-PCR analysis disclosed that the level of HNF4α was significantly reduced in NB cells (Figure 3A,B). Subsequently, we found that HNF4α detetion could markedly impede cell proliferation *in vitro* (Figure 3C,D). At the same time, cell migration and invasion were analyzed in SKNBE-2 and SK-N-SH cells, and MTT analysis exhibited that the abilities of the mobility and invasiveness were evidently restrained *in vitro* (Figure 3E,F). In addition, the alteration of E-cadherin, N-cadherin, and Vimentin indicated that HNF4α silencing distinctly suppressed EMT in NB cells (Figure 3G–J). The evidence displayed that HNF4α worked as an oncogenic role in SKNBE-2 and SK-N-SH cells.

The article "Long non-coding RNA SNHG16 regulates cell behaviors through miR-542-3p/HNF4α axis via RAS/RAF/MEK/ERK signaling pathway in pediatric neuroblastoma cells" was retracted in 2024. Reasons: plagiarized images; duplicated images; overlap with other authors' work; overlap with earlier publications.

**Figure 3:** HNF4α knockdown restrained cell proliferation, migration, invasion, and EMT *in vitro* (**A,B**) qRT-PCR and Western blot assays were performed to confirm the efficiency of si-HNF4α in NB cells. (**C,D**) MTT assay was conducted to expound the role of HNF4α knockdown in cell proliferation *in vitro*. (**E,F**) Cell migration and invasion were assessed utilizing transwell assay. (**G–J**) The level of EMT-relative proteins, including E-cadherin, N-cadherin, and Vimentin, were measured by Western blot. *P<0.05.

### SNHG16 was a sponge of miR-542-3p to isolate HNF4α

Owing to the functions of SNHG16 and HNF4α in NB cells, we searched for the associated factors between SNHG16 and HNF4α. First, the candidate targets of SNHG16 were predicted by starBase v2.0 software. As shown in Figure 4A, we postulated that SNHG16 exerted its role via targeting miR-542-3p. Subsequently, dual-luciferase reporter assay was performed to elucidate whether SNHG16 was a sponge of miR-542-3p, the results clarified that miR-542-3p mimic could distinctly reduce the luciferase activity of WT-SNHG16 reporter, whereas the luciferase activity of mutation had no apparent alteration (Figure 4B,C). Then, the level of miR-542-3p was determined, qRT-PCR analysis suggested that miR-542-3p level was aberrantly down-regulated in NB tissues and cell lines (Figure 4D,E). Furthermore, the level of miR-542-3p was negatively correlated with SNHG16 level (Figure 4F). To consolidate our findings, si-SNHG16 or pcDNA-SNHG16 was transfected into SKNBE-2 and SK-N-SH cells, we found that SNHG16 knockdown could significantly trigger miR-542-3p level, while the up-regulation of SNHG16 specially constrained miR-542-3p level in NB cells (Figure 4G). Similarly, the complementary sequences between miR-542-3p and HNF4α were predicted by starBase v2.0 software, and the results were shown in Figure 4H. Next, miR-542-3p mimic or miR-NC was co-transfected with wild-type or mutant reporter into SKNBE-2 and SK-N-SH cells, respectively. In the dual-luciferase reporter assay, miR-542-3p mimic could induce a decrease in the luciferase activity of HNF4α 3′UTR-WT, but had not evident impact on the mutant reporter of HNF4α 3′UTR-MUT (Figure 4I,J). Meanwhile, miR-542-3p level was passively related to HNF4α level (Figure 4K). Interestingly, miR-542-3p mimic substantially restrained HNF4α level, while the inhibiting role of miR-542-3p up-regulation in HNF4α level was restored via synchronous transfection with pcDNA-SNHG16 in NB cells (Figure 4L,M). In brief, these data discovered that SNHG16 was a sponge of miR-542-3p to regulate HNF4α in NB cells.

The article "Long non-coding RNA SNHG16 regulates cell behaviors through miR-542-3p/HNF4α axis via RAS/RAF/MEK/ERK signaling pathway in pediatric neuroblastoma cells" was retracted in 2024. Reasons: plagiarized images; duplicated images; overlap with other authors' work; overlap with earlier publications.

**Figure 4:** SNHG16 was a sponge of miR-542-3p to isolate HNF4α (**A**) The binding sites between miR-542-4p and SNHG16 were predicted by starBase v2.0. (**B,C**) Dual-luciferase reporter assay was carried out to assay the interaction between miR-542-3p and SNHG16. (**D,E**) The level of miR-542-3p in NB tissues and cell lines was identified. (**F**) qRT-PCR was performed to verify the correlation between miR-542-3p level and SNHG16 level. (**G**) The role of si-SNHG16 and pcDNA-SNHG16 in regulating miR-542-3p level was verified. (**H**) Prediction of the complementary sequences between miR-542-3p and HNF4α were shown. (**I,J**) The relationship between miR-542-3p and HNF4α was clarified using dual-luciferase reporter assay. (**K**) The correlation between miR-542-3p level and HNF4α level was analyzed. (**L,M**) The expression of HNF4α was detected adopting Western blot. *P<0.05.

### The impact of SNHG16 detetion on cell behaviors was regained by HNF4α up-regulation in NB cells

Based on the regulatory mechanism between SNHG16 and HNF4α, si-SNHG16 alone, or along with pcDNA-HNF4α was transfected into SKNBE-2 and SK-N-SH cells. Western blot analysis manifested that the inhibitory effect of SNHG16 knockdown on HNF4α level was recovered after transfection with pcDNA-HNF4α (Figure 5A,B). Then, cell proliferation was examined, and MTT analysis clarified that the inhibiting impact of si-SNHG16 on cell proliferation was reverted after synchronous transfection with pcDNA-HNF4α (Figure 5C,D). At the same time, reintroduction of pcDNA-HNF4α could overturn the suppressive role of SNHG16 silencing on cell migration and invasion in SKNBE-2 and SK-N-SH cells (Figure 5E,F). At last, the expression levels of E-cadherin, N-cadherin, and Vimentin were used to represent the level of EMT in NB cells, Western blot analysis disclosed that SNHG16 detetion could retard EMT, while the curbed effect of SNHG16 deficiency on EMT was regained by up-regulation of HNF4α *in vitro* (Figure 5G–J). In brief, overexpression of HNF4α could abrogate the inhibiting effects of SNHG16 silencing on cell proliferation, migration, invasion, and EMT in NB cells.

**Figure 5:** The impact of SNHG16 detetion on cell behaviors was regained by HNF4α up-regulation in NB cells SKNBE-2 and SK-N-SH cells were transfected with si-NC, si-SNHG16, si-SNHG16+pcDNA, or si-SNHG16+pcDNA-HNF4α, respectively, (**A,B**) and the protein level of HNF4α was estimated via Western blot. (**C,D**) The effects of si-SNHG16 and pcDNA-HNF4α on cell proliferation were measured. (**E,F**) The migrated cells or invaded cells were counted and quantified by transwell assay. (**G–J**) Western blot assay was employed to determine the expression levels of E-cadherin, N-cadherin, and Vimentin. *P<0.05.

The article "Long non-coding RNA SNHG16 regulates cell behaviors through miR-542-3p/HNF4α axis via RAS/RAF/MEK/ERK signaling pathway in pediatric neuroblastoma cells" was retracted in 2024. Reasons: plagiarized images; duplicated images; overlap with other authors' work; overlap with earlier publications.

### Knockdown of SNHG16 could curb the tumor growth *in vivo*

As mentioned before, SNHG16 functioned as an oncogenic gene in NB cells, whether SNHG16 could act the same role *in vivo* was our investigated object. First the stably transfected (lentivirus-mediated sh-SNHG16 or sh-NC) SKNBE-2 cells were injected into nude mice. After the killing of mice, we found that the xenograft tumor volumes and weights were visibly decreased in sh-SNHG16 transfected group than that of sh-NC transfected group (Figure 6A–C). Then, the expression levels of SNHG16, miR-542-3p, and HNF4α were assessed by qRT-PCR, and the results displayed that the levels of SNHG16 and HNF4α were strikingly down-regulated, but miR-542-3p level was notably induced in treatment group (Figure 6D). Simultaneously, the protein expression level of HNF4α was clearly reduced in lentivirus-mediated sh-SNHG16 group (Figure 6E). All the data demonstrated that SHKG16 detetion led to the decrease in NB tumor growth *in vivo*.

**Figure 6:** Knockdown of SNHG16 could curb the tumor growth *in vivo* (**A**–**C**) The tumor volume and weight were recorded and analyzed after mice were killed. (**D**) qRT-PCR was carried out to evaluate the levels of SNHG16, miR-542-3p, and HNF4α in xenograft tumors. (**E**) Western blot was conducted to examine the protein expression level of mature HNF4α in tumor tissues. *P<0.05.

### SNHG16 and HNF4α regulated the development of NB via RAS/RAF/MEK/ERK signaling pathway

Based on the above introductions, we explored whether the RAS/RAF/MEK/ERK signaling pathway went in for the tumorigenic effects of SNHG16 and HNF4α. Then, si-NC, si-SNHG16, si-SNHG16+pcDNA, or si-SNHG16+pcDNA-HNF4α was transfected into SKNBE-2 and SK-N-SH cells, respectively. We observed that SNHG16 detection specifically decreased the level of RAS, p-RAF, p-MEK, and p-ERK in SKNBE-2 cells, while the repressive impact of SNHG16 silencing was abolished after co-transfection with pcDNA-HNF4α (Figure 7A,B). Similar phenomenon occurred in SK-N-SH cells (Figure 7C,D). In summary, SNHG16/miR-542-3p/HNF4α axis regulated NB progression via the activation of RAS/RAF/MEK/ERK signaling pathway (Figure 8).

The article "Long non-coding RNA SNHG16 regulates cell behaviors through miR-542-3p/HNF4α axis via RAS/RAF/MEK/ERK signaling pathway in pediatric neuroblastoma cells" was retracted in 2024. Reasons: plagiarized images; duplicated images; overlap with other authors' work; overlap with earlier publications.

**Figure 7:** SNHG16 and HNF4α regulated the development of NB via RAS/RAF/MEK/ERK signaling pathway Si-NC, si-SNHG16, si-SNHG16+pcDNA, or si-SNHG16+pcDNA-HNF4α was introduced into SKNBE-2 and SK-N-SH cells, respectively. (**A,B**) The level changes of RAS, p-RAF, p-MEK, and p-ERK in SKNBE-2 cells were identified via Western blot assay. (**C,D**) The protein expression level changes of RAS, p-RAF, p-MEK, and p-ERK were detected through Western blot assay in SK-N-SH cells. *P<0.05.

**Figure 8:** SNHG16/miR-542-3p/HNF4α axis regulated NB progression via RAS/RAF/MEK/ERK signaling pathway

## Discussion

In the study, we reported that SNHG16 was highly expressed in NB tissues and cell lines, the deficiency of SNHG16 could obviously constraint several cell behaviors, including cell proliferation, migration, invasion, and EMT in SKNBE-2 and SK-N-SH cells. Before this research, lncRNAs have been suggested to participate in the key events in plenty of tumor processes, might be involved in specific cellular states, including cellular pathologies [24,25]. In addition, the dysregulation of lncRNAs work as the type-specific mechanism in cancers [26]. In regard to SNHG16, the close association between SNHG16 and diverse cancers were reported previously. The high expression of SNHG16 in NB tissues was validated in the present study. Besides, SNHG16 detection could cause the inhibition of cell proliferation, migration, invasion, and EMT in SKNBE-2 and SK-N-SH cells. Furthermore, NB patients with SNHG16 up-regulation had poor overall survival [9]. Apart from that, the oncogenic role of SNHG16 has been reported previously, such as SNHG16 silencing could retard cell growth in gastric cancer [27]. SNHG16 boosted the migration of breast cancer via sponging miR-98 [7]. Currently, emerging evidence exposed that SNHG16 exerted its oncogenic role in glioma tumorigenesis via targeting miR-4518 [28]. However, there were little researches focused on the role of SNHG16 in the pathogenesis and progression of NB.

More and more evidence has displayed that miRNAs are related to largely numerous processes of physiology and pathogenesis [29]. Therefore, we searched for the probable targets of SNHG16, and the bioinformatics software predicted that miR-542-3p had complementary sequences with SNHG16. The dual-luciferase reporter analysis expounded that SNHG16 was a sponge of miR-542-3p in SKNBE-2 and SK-N-SH cells. Then, the decreased expression of miR-542-3p was clarified in NB tissues and cell lines. Not only that, the molecular mechanism between miR-542-3p and SNHG16 was explored, we found that overexpression of SNHG16 could clearly retard miR-542-3p in NB cells. A recent record has indicated that miR-542-3p was highly associated with poor survival of NB patients [20]. Moreover, miR-542-3p functions as a tumor suppressor in several cancers [30]. For instance, Qiao et al. exposed that miR-542-3p restrained the growth of colon cancer, showing as the inhibition of cell migration and invasion in colon cancer cells [31]. Cai et al. indicated that miR-542-3p repressed the capacity of invasion in human astrocytoma via regulating protein kinase B (AKT) signaling pathway [32]. Combining with these findings, we concluded that miR-542-3p was a target of SNHG16 to mediate the progression and initiation in NB.

The article "Long non-coding RNA SNHG16 regulates cell behaviors through miR-542-3p/HNF4α axis via RAS/RAF/MEK/ERK signaling pathway in pediatric neuroblastoma cells" was retracted in 2024. Reasons: plagiarized images; duplicated images; overlap with other authors' work; overlap with earlier publications.

Our present study devotes to understanding the tumorigenesis of NB. Earlier works exhibited that miRNAs can sequester the targeted mRNAs, thereby regulating cellular functions [33]. StarBase v2.0 software revealed that HNF4α was a possible target of miR-542-3p, and the interaction between miR-542-3p and HNF4α was elucidated by dual-luciferase reporter assay. Based on the evidence, we expounded that HNF4α deficiency could constraint cell growth. With regard to the HNF4α, the dysregulation of HNF4α is strictly associated with poor prognosis, metastasis, and dedifferentiation in hepatocellular carcinoma [34]. Some researchers pointed out that HNF4α was frequently observed in advanced lung adenocarcinoma [35], and it could impede the expression of Caudal Type Homeobox 2 (Cdx2), which was a tumor suppressor in intestinal cancer [36]. More importantly, we discovered that overexpression of HNF4α could relieve the repressive role of SNHG16 detetion in cell behaviors. As researched before, RAS/RAF/MEK/ERK signaling pathway inactivation evidently suppressed the progression of hepatocellular carcinoma [22]. Then we measured the corresponding protein expression of this pathway, and the results indicated that SNHG16 could exert its role partially via RAS/RAF/ MEK/ERK signaling pathway.

Taken together, SMHG16 and HNF4α were oncogenic genes, but miR-542-3p could suppress the development of NB. SNHG15 was a sponge of miR-542-3p to separate HNF4α. Functionally, knockdown of SNHG16 or HNF4α distinctly reduced tumor growth in NB cells, showing as the repression of cell proliferation, migration, invasion, and EMT. Importantly, SNHG16 exerted its oncogenic role though miR-542-3p/HNF4α axis via RAS/RAF/MEK/ERK signaling pathway in NB growth. These findings might supply a work pathway of SNHG16 in the progression of NB. However, the limitations in the research should not be neglected, whether SNHG16 can be applied as the biomarker of NB diagnosis requires more evidence.

## Abbreviations

EMT: epithelial–mesenchymal transition
GAPDH: glyceraldehyde-3-phosphate dehydrogenase
HEK293: human embryonic kidney 293
HNF4α: hepatocyte nuclear factor 4 α
lncRNA: long non-coding RNA
miRNA: microRNA
MTT: 3-(4,5-dimethylthiazol-2-yl)-2,5-diphenyl-tetrazolium bromide
NB: neuroblastoma
ncRNA: non-coding RNA
qRT-PCR: quantitative real-time polymerase chain reaction
siRNA: small interfering RNA
SNHG16: small nucleolar RNA host gene 16
